The article "Clinical Comparison of Endoscopic Ultrasonography and CT in Preoperative TN Staging of Esophagogastric Junction Cancer" was retracted in 2023. Reasons: unreliable results or conclusions; lack of ethics approval or compliance; concerns about the data; concerns about the peer review.

# Clinical Comparison of Endoscopic Ultrasonography and CT in Preoperative TN Staging of Esophagogastric Junction Cancer

**DOI:** 10.1155/2022/5810405

**Published:** 2022-09-07

**Authors:** Tao Peng, Zhan Lou, Xiaoyuan Wang, Di Huang, Guiyun Zhang, Huibin Gao, Shuguang Li

**Affiliations:** The First Affiliated Hospital of Hebei North University, Zhangjiakou 075000, Hebei, China

## Abstract

In recent years, the incidence of esophagogastric junction cancer has increased year by year. It is a special type of gastric cancer, with 80% of patients being clinically in the middle and late stages. The traditional treatment methods are extremely ineffective, and the accuracy of preoperative staging is not good enough. At present, the medical treatment for esophagogastric junction cancer mainly adopts surgery and postoperative adjuvant therapy. The current mainstream clinical diagnostic methods of esophagogastric junction cancer before concurrent neoadjuvant chemoradiotherapy are X-ray, CT examination, and gastroscopic diagnosis. However, these clinical diagnostic methods have many limitations. Endoscopic ultrasonography (EUS) can accurately locate malignant tumors in the digestive tract, surrounding microstructures. It can diagnose lymphatic metastasis so as to provide a clear imaging basis for neoadjuvant chemoradiotherapy. This method can also effectively improve the prognosis of the esophagus and stomach according to the characteristics of the patient. In this experiment, we conducted a controlled trial on patients with stage III esophagogastric junction cancer, divided into an experimental group (neoadjuvant chemotherapy + surgery) and a control group (conventional surgery). The preoperative EUS staging in the control group, the preoperative EUS staging in the neoadjuvant chemoradiotherapy group, and the postoperative pathological staging were compared. The experiment showed that in the control group, the preoperative and postoperative accuracy of EUS was 89.2%, while the preoperative and postoperative accuracy of CT examination was only 62.5%. In the experimental group, the preoperative and postoperative accuracies of EUS and CT were 79.6% and 56.7%, respectively. EUS has both specificity and accuracy due to CT examination. Through studying EUS technology in the staging and diagnosis of esophagogastric junction cancer, the therapeutic effect of esophagogastric junction cancer can be improved. The prognosis of esophagogastric junction cancer can also be improved.

## 1. Introduction

The accelerated pace of life, long-term improper diet, and bad living habits lead to an increasing incidence of gastric cancer. Esophagogastric junction cancer is the most common case of gastric cancer. Because most of the clinical manifestations of esophagogastric junction cancer are in the middle and late stages, the traditional radical resection of esophagogastric junction cancer has a very low success rate. With the development of medical industry, the advent of many new anticancer drugs and new programs has a positive impact on the treatment and improvement of prognosis of esophagogastric junction cancer. Neoadjuvant chemotherapy is effective against esophagogastric junction cancer. A regimen of paclitaxel + carboplatin (TP single-week regimen) has good effect and low side effects in chemotherapy of advanced esophagogastric junction cancer. It can be used as the preferred option for preoperative neoadjuvant therapy. However, the traditional preoperative diagnosis mostly adopts CT examination, X-ray, and other methods. The observation of surrounding structures is not accurate enough. Endoscopic ultrasonography is a very valuable tool for diagnosing and TNM staging of gastrointestinal tumors. The outer diameter of the apex of the ring-scan endoscopic ultrasound is 13.8 mm, and the outer diameter of the small ultrasonic probe is 2.5 mm. When the tumor invades the esophageal cavity to form a stenosis, the small ultrasonic probe is often more advantageous, but it is at a disadvantage in the deep ring scan. It is of great significance to select appropriate endoscopic ultrasonography for operation, diagnosis and treatment, and clinical staging before and after concurrent neoadjuvant chemoradiotherapy for esophagogastric junction cancer.

In the face of esophagogastric junction cancer, many researchers have studied the preoperative TN staging of esophagogastric junction cancer by neoadjuvant chemotherapy. Among them, Sos et al., through the study of esophagogastric junction cancer, said that neoadjuvant chemotherapy has more advantages than traditional clinicopathological methods in improving patients and prognosis [1]. Rodica et al. conducted a statistical study of staging patients with esophagogastric junction cancer. They also used different staging patterns for TNM to treat different patients [2]. The study of Laxague et al. pointed out that neoadjuvant chemotherapy is a way to shrink the tumor and remove tumor cells to treat esophagogastric junction cancer [3]. Minami et al. performed preoperative TN staging for patients. After 5 courses of radiotherapy and chemotherapy, the patient's lymph nodes were significantly reduced [4]. Meng et al. compared the method of neoadjuvant chemotherapy and surgery by CT examination with ordinary surgery. It was concluded that the former can effectively improve the treatment effect of esophagogastric junction cancer [5]. Although preoperative TN staging of neoadjuvant chemotherapy has a positive therapeutic effect on esophagogastric junction cancer, there is a lack of methods to precisely observe tumor cells.

Endoscopic ultrasonography can accurately observe cancer cells. This method can also diagnose lymphocyte metastasis. Therefore, many researchers use endoscopic ultrasonography to study preoperative TN staging of esophagogastric junction cancer. Among them, Tanaka et al. used endoscopic ultrasonography to observe cancer cells in a patient with esophagogastric junction cancer, which was successfully removed [6]. Hosoda et al. successfully resected patients with esophagogastric junction cancer through endoscopic ultrasonography, where the operation time was shorter than traditional operation and the patients recovered after surgery [7]. Nagami et al. indicated that endoscopic ultrasonography has a high guiding significance in preoperative TN staging of esophagogastric junction cancer [8]. When Sugita et al. treated an elderly patient with esophagogastric junction cancer, the patient's condition was controlled by changing the staging time of radiotherapy and chemotherapy [9]. Zhang et al.' clinical analysis of esophagogastric junction cancer revealed that neoadjuvant therapy with endoscopic ultrasonography can improve the resection rate of cancer cells [10]. The ability of endoscopic ultrasonography to accurately observe cells can greatly help the preoperative TN staging analysis of esophagogastric junction cancer, but it has not been compared with CT examination and other methods.

In this paper, a clinical comparison of endoscopic ultrasonography and CT examination in preoperative TN staging of esophagogastric junction cancer is carried out. The innovations are summarized in the following aspects: (1) selecting ring-scan endoscopic ultrasonography and small ultrasonic probe in the diagnosis of esophagogastric junction cancer with different degrees of stenosis; (2) comparing TNM staging and postoperative pathological staging of endoscopic ultrasonography after neoadjuvant chemorotherapy for esophagogastric junction cancer; (3) establishing an imaging evaluation model for evaluating the effect of comprehensive treatment of esophagogastric junction cancer, and formulating a diagnosis and treatment plan based on the characteristics of patients.

## 2. Ultrasound Endoscopy and CT Examination Methods

Esophagogastric junction cancer is a kind of adenocarcinoma, which is mainly caused by the canceration of gastric mucosa cells, because the source of the disease comes from the gastric mucosa. The process of esophagogastric junction cancer diagnosis is shown in Figure 1. In the process of esophagogastric junction cancer diagnosis, influence detection and screening constitute a very important step. It is difficult for ordinary detectors to accurately observe the source of the disease. At present, the mainstream methods for detecting esophagogastric junction cancer are endoscopic ultrasonography and CT examination [11].

### 2.1. Endoscopic Ultrasonography

#### 2.1.1. Principle of Endoscopic Ultrasound Imaging

Ultrasound imaging is one of the important ways of medical image screening, and its principle is to transmit medical information through ultrasound. It mainly uses its echo information between human tissues to analyze the echo information for medical diagnosis [12]. In the process of ultrasonic transmission of information, the closely related parameters are ultrasonic frequency, ultrasonic propagation speed, ultrasonic reflection and refraction, and ultrasonic propagation weakening.

*(1) Ultrasonic frequency*. Ultrasound is a kind of sound wave. The frequency of sound wave is between 10^−4^ Hz and 10^14^ Hz. The sound wave with frequency higher than 20000 Hz is called ultrasonic wave. Ultrasound used in medical imaging procedures is between 5 MHz and 35 MHz. Generally, the ultrasonic frequency selected is different according to the different parts to be detected. In general, the higher the ultrasound frequency is, the higher the detection resolution will be. However, the lower the ultrasound frequency is, the worse the detection resolution will be, but the greater the depth and breadth will be [13].

*(2) Ultrasonic propagation speed*. The speed of sound wave propagation is affected by the medium. In general, the speed of propagation in solids is better than that in liquids, while the speed of propagation in liquids is better than that in gases. Ultrasound also follows this principle. More than 70% of the human body is composed of water, so the propagation speed of ultrasonic waves in the human body is as in the following formula:

(1) $$\begin{array}{c} C=\mu \times g. \end{array}$$

In (1), *C* represents the propagation speed of ultrasonic waves in the human body, *μ* represents the wavelength, and *g* represents the frequency of the sound wave.

Due to the different components of different parts of the human body, the propagation speed of ultrasonic waves in different tissues of the human body will also be different. Therefore, as long as the propagation speed of ultrasonic waves in various tissues of the human body is clear, the distance between human tissues in medical treatment can be well calculated. The propagation speed of ultrasonic waves between various tissues of the human body is shown in Table 1.

*(3) Reflection and refraction of ultrasonic waves*. Ultrasonic waves have the same characteristics as sound waves. Reflection and refraction will occur when they are transmitted at the junction of the two media. The schematic diagram of refraction and reflection is shown in Figure 2. In Figure 2, the incident wave is denoted by *α*_1_. The reflected wave is denoted by *α*_2_, and the transmitted wave is denoted by *α*_3_. Among them, medium 1 is represented by *μ*_1_, and the speed in medium 1 is *c*_1_; medium 2 is represented by *μ*_2_, and the speed in medium 2 is *c*_2_.

Then the resistance in medium 1 is as follows:

(2) $$\begin{array}{c} Q_{1}=\mu_{1}c_{1}. \end{array}$$

The resistance in medium 2 is as follows:

(3) $$\begin{array}{c} Q_{2}=\mu_{2}c_{2}. \end{array}$$

The relationship between the angle of incidence, the angle of reflection, and the angle of transmission is expressed by the following formulas:

(4) $$\begin{array}{c} \theta_{1}=\theta_{2}. \end{array}$$

(5) $$\begin{array}{c} \frac{\sin\theta_{1}}{\sin\theta_{3}}=\frac{c_{1}}{c_{3}}. \end{array}$$

In medical imaging, ultrasonic waves are generally incident on human tissue vertically to obtain the maximum reflected ultrasonic waves. Due to the different reflectivity of human tissues, the reflectivity of ultrasonic waves in human tissues is shown in Table 2.

*(4) Weakness of ultrasound transmission*. In the process of ultrasonic propagation, its sound wave intensity and amplitude will be reduced by the interference of physical factors such as the propagation medium, which is the process of ultrasonic propagation weakening [14].

According to the principle of ultrasonic propagation, the echo of ultrasonic wave is expressed as follows:

(6) $$\begin{array}{c} H\left(t\right)=A\left(x\right)I_{0}e^{2bx}=A\left(x\right)I_{0}e^{2\text{bct}}. \end{array}$$

In (6), *A*(*t*) represents the ultrasonic echo information, *b* is the weakening parameter of the human body, *A*(*x*) represents the reflection, *I*_0_ represents the intensity of the ultrasonic wave when it is emitted, *c* represents the ultrasonic wave propagation speed in the human body, and *t* represents the propagation time.

*H*(*t*) in formula (6) is exponentially related to the attenuation decibel number. Then, the following formula can be obtained:

(7) $$\begin{array}{c} H_{DB}=20\mathrm{lg}H\left(t\right)=rt+d. \end{array}$$

It can be seen from (7) that *r* and *d* are constants and the attenuation decibel number *H*_*DB*_ of the ultrasonic wave has a linear relationship with the propagation time *t*. Therefore, in the actual application of medical imaging, it is necessary to perform weakening compensation on the ultrasonic echo information, so that accurate and specified ultrasonic echo information can be obtained.

#### 2.1.2. Principle of Phase-Controlled Ultrasonic Imaging

*(1) Principle of phased array propagation*. The phased array is to control the propagation time between the array units, so that it can be focused at any place. Then, precise control of the ultrasonic wave can be achieved. The phased array is divided into a transmitting end and a receiving end. At the transmitting end, if the two outer array units transmit inwards first, ultrasonic focusing will occur. If each array unit transmits at the same angle, the ultrasonic deflection phenomenon will occur, which is the principle of ultrasound endoscopic imaging.

The receiving end of the phased array is determined by the time when each array unit receives the signal. After a series of compensation measures, the demultiplexed waves are synthesized. The principle of the receiving end of the phased array is shown in Figure 3.

*(2) Principle of relative delay*. The basis of the working principle of ultrasonic phased array is relative delay, which is the principle that the focused or scattered ultrasonic information of each array unit is different. The relative delay can be used to achieve precise control of the ultrasonic beam and improve the quality of ultrasonic imaging [15].

The principle of relative delay is shown in Figure 4. When the number of array elements is odd, the center of the array is at 0. When the number of elements is even, the center of the array is between 0 and 1.

As can be seen from Figure 4, the distance from point P to any array unit is as follows:

(8) $$\begin{array}{c} D_{n}=\sqrt{{\left(l\cos\theta \right)}^{2}+{\left(l\sin\theta -\left(n-\frac{1}{2}\right)l\right)}^{2}}. \end{array}$$

In (8), *l* represents the vertical distance from P to the probe, *n* represents the number of array elements, and cos is the cosine function.

Then, the delay from the array unit to 0 can be expressed as follows:

(9) $$\begin{array}{c} \phi_{n}=\frac{D_{n}-l}{c}. \end{array}$$

In (9), *c* is the ultrasonic wave propagation velocity.

Generally, improving the accuracy of the relative delay can improve the imaging quality of the entire ultrasound system. The accuracy of the relative delay directly affects the beam side error. The ratio *S* between the beam side error and the beam amplitude is expressed as follows:

(10) $$\begin{array}{c} S=\sqrt{\frac{1-\sin c\left(1/\lambda \right)}{N\sin c\left(1/\lambda \right)}}\approx \frac{\pi }{\lambda {\left(6N\right)}^{1/2}}. \end{array}$$

In (10), *λ* is the product of the ultrasonic center frequency and the precision, *N* represents the number of array elements, and sin is a sine function.

(11) $$\begin{array}{c} \sin c\left(s\right)=\frac{\sin\pi s}{\pi s}. \end{array}$$

Therefore, when the relative delay accuracy is improved or the number of array units is increased, the clarity of ultrasonic imaging can be improved.

### 2.2. CT Examination Technology

#### 2.2.1. Principle of CT Imaging

CT examination is a type of computed tomography examination, which is a common medical examination method without harming the human body. The imaging principle of CT inspection is essentially a process of converting electrical signals into digital signals, which are then processed by computers and other equipment to present an image of human body structure [16].

The basic principles of CT imaging and X-ray are the same, both of which are used to observe the ability of different parts of the human body to absorb light. The image with strong light absorption ability will appear as bright white or gray on the image, while the weak absorption ability will appear as blackish on the image. CT examination can be very good for the clear detection of human soft tissue or gastrointestinal tissue. The model of CT examination is shown in Figure 5.

#### 2.2.2. Principle of Ant Colony Algorithm

Due to the high complexity of CT images, different tissues may show different gray levels in the same CT image. They also include a lot of impurity information such as noise. Therefore, it is very important to process CT images. Using the ant colony algorithm, the pixels in the image can be regarded as the pheromone in the algorithm. Under the ant colony algorithm, the edges of CT images can be found quickly and accurately, through which medical images can be clearly presented [17].

Using the ant colony algorithm, the set of image pixels to be traversed is set to *B*={*b*_1_, *b*_2_, ⋯, *b*_*n*_}, and the set of connections between two pixels is represented by *L*={*l*_*ij*_*|b*_*i*_, *b*_*j*_ ∈ *B*}. The distance between two pixels is represented by *r*_*ij*_(*i*, *j*=1,2, ⋯, *n*).

Then, the formula for *r*_*ij*_ is expressed as equation 12.

The detection of CT images is to traverse all the pixels in the image, and each pixel can only be traversed once [18]. Assuming that the number of ants in the *i*th pixel at time *t* is *m*_*i*_(*t*), the total number of ants is *Sum*=∑_*i*=1_^*n*^*m*_*i*_(*t*), and the pheromone left between two pixels *i* and *j* at time *t* is Msg_ij_(*t*). Then, from time *t* to time *t* + 1, when each ant passes a pixel point, the pixel pheromone will be updated. The formula is expressed as follows:

(12) $$\begin{array}{c} {\text{Msg}}_{\text{ij}}\left(1+t\right)=\left(1-\rho \right)\cdot {\text{Msg}}_{\text{ij}}\left(t\right)+\Delta {\text{Msg}}_{\text{ij}}. \end{array}$$

In (12), *ρ* represents the pheromone factor.

The change amount ΔMsg_ij_ of pheromone is expressed as follows:

(13) $$\begin{array}{c} \Delta {\text{Msg}}_{\text{ij}}=\sum_{k=1}^{m}\Delta {\text{Msg}}_{ij}^{k}. \end{array}$$

In (13), ΔMsg_ij_^*k*^ represents the pheromone left between the pixel points *i* and *j* when the *k*-th ant changes from time *t* to time *t* + *n*. The formula is expressed as follows:

(14) $$\begin{array}{c} \Delta {\text{Msg}}_{\text{ij}}^{k}=\left\{\begin{array}{cc} \frac{R}{r_{k}}, & \left(t,t+n\right)⟶\left(i,j\right),\\ 0\text{,} & \text{other}. \end{array}\right.. \end{array}$$

In (14), *R* is a constant, and *r*_*k*_ is the distance of the pixels that the ants traveled this time. represents the amount of change in time.

According to the pheromone left by the ants at different pixel points in time, the probability value can be calculated. That is, the probability of ant *k* changing from pixel *i* to pixel *j* at time *t* is expressed as follows:

(15) $$\begin{array}{c} P_{ij}^{k}=\left\{\begin{array}{cc} \frac{{\left[{\text{Msg}}_{\text{ij}}\left(t\right)\right]}^{a}.{\left[\sigma_{ij}\right]}^{b}}{\sum_{k\in {\text{allowed}}_{k}}{\left[{\text{Msg}}_{\text{ik}}\left(t\right)\right]}^{a}.{\left[\sigma_{ij}\right]}^{b}}, & \text{if}\left(j\in {\text{alowed}}_{k}\right),\\ 0, & \text{other}. \end{array}\right. \end{array}$$

In (15), *k* ∈ *allowed*_*k*_ represents the pixels that the *k*-th ant can choose, *a* represents the route optimization factor, *b* represents the expectation factor, and *σ*_*ij*_(*t*) represents the expectation function.

Among them, *σ*_*ij*_(*t*) expectation function can be expressed as follows:

(16) $$\begin{array}{c} \sigma_{ij}\left(t\right)=\frac{1}{r_{ij}}. \end{array}$$

In (16), *r*_*ij*_ represents the distance from *i* to *j*.

The principle of ant colony algorithm is to update the probability of state transition and know to find an optimal solution. Its algorithm flow is shown in Figure 6.

The update of the pheromone of the ant colony algorithm is the core of the algorithm. Formula (14) is only one of them. The other ways to update the pheromone are as in the following formulas:

(17) $$\begin{array}{c} \Delta {\text{Msg}}_{ij}^{k}=\left\{\begin{array}{cc} \frac{R}{r_{ij}}, & \left(t,t+1\right)⟶\left(i,j\right),\\ 0, & \text{other}. \end{array}\right. \end{array}$$

In (17), *R* is a constant.

(18) $$\begin{array}{c} \Delta {\text{Msg}}_{ij}^{k}=\left\{\begin{array}{cc} R, & \left(t,t+1\right)⟶\left(i,j\right),\\ 0, & \text{other}. \end{array}\right. \end{array}$$

Formulas (17) and (18) are a local pheromone optimization method. Pheromone is left after every time a pixel is passed, and it is not necessary to go through all the pixels. But in solving complex optimization problems such as CT examination, the algorithm of (14) is better.

## 3. Clinical Trial of Endoscopic Ultrasonography and CT in Preoperative TN Staging of Esophagogastric Junction Cancer

### 3.1. Experimental Data

#### 3.1.1. Data Sources

In order to better compare the clinical manifestations of endoscopic ultrasonography (EUS) and CT in preoperative TNM staging of esophagogastric junction cancer, this experiment selected gastroscopic biopsy for pathological diagnosis between 2016 and 2021. Using EUS staging, 60 patients with stage III esophagogastric junction cancer were diagnosed [19].

The criteria for the inclusion of patients were as follows: The patients themselves were unaware of the experiment and had never received any anticancer drugs or other drugs. The patients were diagnosed with stage III esophagogastric junction cancer. All imaging data should be complete. The patients had no other cardiopulmonary diseases, with physical fitness score KPS >70 and age <75 years old. The exclusion criteria were as follows: patients who refused to be enrolled in clinical research; patients with contraindications to treatment; patients who had special circumstances during the treatment process, or patients who could not complete the treatment due to the toxic and side effects of the treatment; patients who were older than 75 years old [20].

This experiment will be divided into two parts. In the experimental group (neoadjuvant chemoradiotherapy group), 30 patients with stage III esophagogastric junction cancer were given TP regimen (paclitaxel + carboplatin) neoadjuvant chemotherapy for 1 week and then given concurrent radiotherapy for 4 days. At the same time, neoadjuvant chemotherapy was given until 4 weeks after the radiotherapy was stopped, and endoscopic ultrasound staging was performed again before surgery, with 3-week rest. Then, the surgery was performed.

  For chemotherapy in the experimental group, TP regimen (paclitaxel: 80 mg/m^2^, carboplatin AUC 1.5, once a week, totally 8 weeks) was given. Surgery began after 3 weeks of rest.
  For radiotherapy in the experimental group, linear accelerator 6 MV X-ray, CT localization, and three-dimensional conformal intensity-modulated radiotherapy were used. The dose of radiotherapy was 40 Gy/20 F/4 W.
  In the control group (conventional operation group), 30 patients with stage III esophagogastric junction cancer were directly treated with radical resection of esophagogastric junction cancer [21].

The basic information of the experimental participants is shown in Table 3.

#### 3.1.2. Evaluation Criteria for Endoscopic Ultrasonography of Primary Tumors

The staging of esophagogastric junction cancer was divided into two types, uT staging and uNM staging.The evaluation criteria for staging are shown in Table 4.

### 3.2. Comparison of Preoperative uTNM Staging and Postoperative Pathological Staging in the Control Group

The medical diagnosis and treatment steps of the control group were as follows: 30 patients with stage III esophagogastric junction cancer (pathology, endoscopic ultrasonography, CT imaging evaluation) ⟶ routine operation group (radical resection of esophagogastric junction cancer) ⟶ CT examination, EUS staging compared with postoperative pathological staging [22].

In order to fully compare the preoperative uTNM staging results of CT and EUS, the sensitivity, specificity, and accuracy of preoperative uTNM staging and postoperative pathological staging were compared and analyzed.

#### 3.2.1. Sensitivity Analysis

Because most cases of esophagogastric junction cancer are found in the middle and late stages and the treatment is difficult, the clinical analysis of the patients is very important for the later treatment. The sensitivity of preoperative staging determines the initial time of preoperative staging. The comparison results of preoperative staging sensitivity for 30 patients with stage III esophagogastric junction cancer are shown in Figure 7.

From the analysis of Figure 7, it can be seen that in the preoperative uT staging, the sensitivity of uT3 in the period with the best EUS sensitivity was 84.5%, while the sensitivity of uT4a in the period with the best CT sensitivity was 82.8%. In preoperative uNM staging, EUS had the best sensitivity in period N1 with a sensitivity of 85.9%, while CT had the best sensitivity in period N1 with a sensitivity of 81.3%.

#### 3.2.2. Specificity Analysis

Analysis of the specificity of esophagogastric junction cancer can be a good solution to the patient's condition. The comparison results of preoperative staging specificity of 30 patients with stage III esophagogastric junction cancer are shown in Figure 8.

From the analysis of Figure 8, it can be seen that the difference between EUS specificity and CT specificity in preoperative uT staging was not very large. But in preoperative uNM staging, EUS specificity and CT specificity were very different. Among them, the average specificity of EUS for nNM was 85.7%.

#### 3.2.3. Accuracy Analysis

The accuracy of preoperative staging of esophagogastric junction cancer compared with postoperative pathological staging is the most important step in staging and treating patients. The accuracy of preoperative staging can not only maximize the optimal treatment time for patients, but also improve the treatment efficiency of patients.  Figure 9 shows the comparison results of preoperative staging accuracy for 30 patients with stage III esophagogastric junction cancer.

From the analysis of Figure 9, it can be seen that, whether it was preoperative uT staging or uNM staging, the staging accuracy of EUS was higher than that of CT staging. The average accuracy of uT staging was higher than that of uNM. Among them, the highest accuracy of EUS in uT staging was 95.9% of uT3, while the highest accuracy of EUS in uNM staging was 91.8% of N0.

### 3.3. Comparison of Preoperative uTNM Staging and Postoperative Pathological Staging in Neoadjuvant Chemoradiotherapy Group

The medical diagnosis and treatment steps of the experimental group were as follows: 30 patients with stage III esophagogastric junction cancer (pathology, endoscopic ultrasonography, CT imaging evaluation) → neoadjuvant chemotherapy group (TP regimen for 9 weeks) → CT examination, EUS staging and postoperative pathological staging comparison.

Similarly, the sensitivity, specificity, and accuracy of preoperative uTNM staging and postoperative pathological staging were compared on CT and EUS preoperative uTNM staging results.

#### 3.3.1. Sensitivity Analysis

Thirty patients with stage III esophagogastric junction cancer in the neoadjuvant chemoradiotherapy group underwent CT preoperative staging and EUS staging. By comparison with postoperative pathological staging, the advantages and disadvantages of the two methods of preoperative staging in neoadjuvant chemoradiotherapy were discussed. The comparison results of preoperative staging sensitivity of patients are shown in Figure 10.

From the analysis of Figure 10, it can be seen that in the neoadjuvant chemoradiotherapy group, the sensitivity of EUS preoperative staging has reached a very high level. The sensitivity of EUS preoperative staging in Figure 10(a)was 76.3% on average, while the sensitivity of EUS preoperative staging in Figure 10(b)was 75.6% on average. The sensitivity of CT preoperative staging was not much different from that in the control group. The sensitivity of CT preoperative staging in Figure 10(a) was 70.0% on average, and the sensitivity of CT preoperative staging in Figure 10(b) was 74.1% on average.

#### 3.3.2. Specificity and Accuracy Analysis

The specificity and accuracy of preoperative staging are the indicators that can best reflect the treatment effect of patients with esophagogastric junction cancer. The patients in the neoadjuvant chemotherapy group were subjected to CT preoperative staging, EUS staging, and then the above-mentioned radiotherapy and chemotherapy courses. By comparing the preoperative staging and postoperative pathological staging, the advantages and disadvantages of the two preoperative staging types under the neoadjuvant chemotherapy mode were discussed [23]. The comparison results of preoperative staging specificity and accuracy of patients are shown in Figure 11.

From the analysis of Figure 11, it can be seen that the specificity of EUS preoperative staging in the neoadjuvant chemotherapy group in Figure 11(a) was better than that of CT preoperative staging. Among them, the average specificity of EUS preoperative staging was 79.0%, while the average specificity of CT preoperative staging was 72.2%. The EUS preoperative staging accuracy in the neoadjuvant chemotherapy group in Figure 11(b) was also better than that of CT preoperative staging. Among them, the average accuracy of EUS preoperative staging was 79.6%, while the average accuracy of CT preoperative staging was 56.7%.

### 3.4. Experimental Results

The patients with stage III esophagogastric junction cancer were treated by comparing conventional radical resection and neoadjuvant concurrent chemoradiotherapy. CT and EUS preoperative staging were used in the treatment to compare the sensitivity, specificity, and accuracy of the two preoperative uTNM staging types and the postoperative pathological staging. The results of the mean difference between the preoperative uTNM staging and postoperative pathological staging of the experiment are shown in Table 5.

## 4. Discussion

The incidence of esophagogastric junction cancer is increasing year by year, and its treatment effect is often poor. We used endoscopic ultrasonography and CT examination to evaluate the accuracy of preoperative uTNM and postoperative pathological staging of neoadjuvant chemotherapy (paclitaxel + carboplatin) for esophagogastric junction cancer so that accurate medical imaging evidence for clinical treatment of esophagogastric junction cancer can be provided.

## 5. Conclusions

Through the clinical comparative experimental analysis of EUS and CT in preoperative uTNM staging of esophagogastric junction cancer, the following conclusions are drawn: (1) In ordinary radical resection of esophagogastric junction cancer, the average sensitivity, specificity, and accuracy of EUS preoperative staging are 80.2%, 88.4%, and 89.2%, respectively, which performs better than CT preoperative staging; (2) EUS in the neoadjuvant chemotherapy mode had an average sensitivity of 0.7%, an average specificity of 6.3%, and an average accuracy of 22.9% better than that of CT for preoperative staging; (3). The neoadjuvant chemotherapy group had similar sensitivity, specificity, and accuracy as the conventional surgery group. Therefore, endoscopic ultrasonography is suitable for staging evaluation after neoadjuvant chemotherapy. The experimental comparison of EUS and CT pathology before and after surgery is based on three aspects: sensitivity, specificity, and accuracy. However, more dimensions are required for comparison to fully analyze the clinical comparison of preoperative staging between the two methods, which will be the direction of future research.

## Figures and Tables

**Figure 1:** Flowchart of the diagnosis of esophagogastric junction cancer.

**Figure 2:** Ultrasonic reflection and refraction diagram.

**Figure 3:** Schematic diagram of the phased array receiver.

**Figure 4:** Schematic diagram of relative delay.

**Figure 5:** Model diagram of CT examination.

**Figure 6:** Flowchart of ant colony algorithm.

**Figure 7:** Sensitivity comparison results of preoperative staging in conventional surgery. (a) uT staging sensitivity. (b) uNM staging sensitivity.

**Figure 8:** Comparison of preoperative staging specificity of conventional surgery. (a) uT staging specificity. (b) uNM staging specificity.

**Figure 9:** Comparison of the accuracy of preoperative staging in conventional surgery. (a) uT staging accuracy. (b) uNM staging accuracy.

**Figure 10:** Sensitivity comparison of preoperative staging for neoadjuvant chemoradiotherapy. (a) uT staging sensitivity. (b) uNM staging sensitivity.

**Figure 11:** Comparison of the specificity and accuracy of preoperative staging of neoadjuvant chemoradiotherapy. (a) Preoperative staging specificity. (b) Preoperative staging accuracy.

**Table 1:** Propagation velocity table of ultrasonic waves between various tissues of the human body.

Human tissue	Transmission speed	Characteristic impedance (kgm^−2^s^−1^)
Blood	1570 m/s	1.60 × 10^6^
Brain tissue	1540 m/s	1.59 × 10^6^
Fat	1540 m/s	1.39 × 10^6^
Liver	1550 m/s	1.65 × 10^6^
Muscle	1590 m/s	1.71 × 10^6^
Skull	4000 m/s	7.79 × 10^6^
Soft tissue	1540 m/s	1.62 × 10^6^

**Table 2:** Reflectance table of ultrasound in human tissue.

The junction of different tissues in the human body	Vertical reflectivity
Muscle and liver	0.02
Muscles and kidneys	0.03
Muscle and blood	0.04
Fat and kidneys	0.07
Soft tissue and blood	0.04
Bone and fat	0.70
Skull and brain	0.67
Fat and liver	0.08

**Table 3:** Basic information of the participants in the experiment.

Baseline data	Surgery group (*n* = 30)	Chemotherapy group (*n* = 30)
Gender{*n*(%)}		
Male	22(73.3%)	20(66.7%)
Female	8(26.7%)	10(33.3%)
Age {(*X*±*S*)years}	61.867 ± 8.11	60.100 ± 7.96
Weight {(*X* ± *S*)kg}	64.167 ± 9.70	62.267 ± 9.13
Height {(*X* ± *S*)cm}	168.600 ± 8.85	165.133 ± 9.12
Clinical TNM stage {*n*(%)}		
T3N0M0	0(0%)	1(3.3%)
T3N1M0	10(33.3%)	7(23.3%)
T3N2M0	3(10.0%)	4(13.3%)
T3N3M0	2(6.7%)	4(13.3%)
T4aN0M0	0(0%)	2(6.7%)
T4aN1M0	7(23.3%)	6(20.0%)
T4aN2M0	6(20.0%)	5(16.7%)
T4aN3M0	2(6.7%)	1(3.3%)

**Table 4:** Evaluation criteria for endoscopic ultrasonography of primary tumors.

uT staging	uNM staging
uT1a: invasion of the mucosal layer	N0: no lymph node metastasis
uT1b: invasion of the submucosa	N1: 1-2 lymph node metastasis
uT2: violation of the muscularis propria	N2: 3-6 lymph node metastases
uT3: invasion of connective tissue	N3: 7 or more lymph node metastases
uT4a: invasion of the visceral peritoneum	M0: no distant metastases
uT4b: violation of peripheral organs	M1: there is distant metastasis

**Table 5:** Preoperative uTNM staging and postoperative pathological staging table.

Staging method	Control group			Test group		
	Sensitivity (%)	Specificity (%)	Accuracy (%)	Sensitivity (%)	Specificity (%)	Accuracy (%)
EUS	80.2	88.4	89.2	75.8	79.0	79.6
CT	78.5	80.9	62.5	75.1	72.7	56.7

## Data Availability

The data that support the findings of this study are available from the corresponding author upon reasonable request.
